The article "Treatment of Cancer Gene Changes in Chronic Myeloid Leukemia by Big Data Analysis Platform-Based Dasatinib" was retracted in 2023. Reasons: signs of a paper mill; compromised peer review; unreliable results or conclusions.

# Treatment of Cancer Gene Changes in Chronic Myeloid Leukemia by Big Data Analysis Platform-Based Dasatinib

**DOI:** 10.1155/2022/9294634

**Published:** 2022-06-10

**Authors:** Linlin Song, Qi Li, Hui Shi, Pengxia Zhang

**Affiliations:** ^1^School of Basic Medicine, Jiamusi University, Jiamusi, 154007 Heilongjiang, China; ^2^Department of Biochemistry, Mudanjiang Medical School, Mudanjiang, 157011 Heilongjiang, China; ^3^Department of Pharmacy, First Affiliated Hospital of Jiamusi University, Jiamusi, 154007 Heilongjiang, China

## Abstract

Based on data mining, an innovative big data analysis platform was utilized to discuss the treatment of cancer in chronic myeloid leukemia (CML) by dasatinib, aiming to offer help to the diagnosis and treatment of cancer. An integrated gene expression analysis system (IEAS) was firstly constructed to automatically classify data in the online human Mendelian genetic database using clustering algorithms. At the same time, the gene expression profile was analyzed by principal component analysis (PCA) in the analysis system. In addition, the efficacy of dasatinib in the treatment of patients with advanced CML was then retrospectively analyzed. The results showed that the IEAS system could incorporate the gene expression analysis vectors it contained by JAVA-related technologies, and the generated clustering genes showed similar functions. The clustering algorithm could homogenize data and generate visual clustering heat maps. The analysis results of major elements were diverse under different experimental conditions. The characteristic value of the first major element was the largest. Messenger ribonucleic acid (mRNA) datasets of CML patients were selected from cancer genomic map, including 120 samples and 20,614 mRNA in total. In micro-RNA (miRNA) datasets, there were 202 samples including 1,406 miRNAs. Data were screened by miRNA–mRNA regulation template, and 20 differentially expressed mRNAs were obtained. In conclusion, the proposed IEAS system could mine and analyze the gene expression data. Dasatinib showed good efficacy in the treatment of patients with advanced CML. Besides, it could improve visual queries, and data mining had a broad application prospect in clinical application. Dasatinib was considered to be a good option for patients with advanced CML.

## 1. Introduction

Chronic myeloid leukemia (CML) is a relatively rare disease caused by malignant tumor and a malignant clonal disease originating from hemopoietic stem cells. It accounts for about 0.3% of all malignant tumors and 20% of adult leukemia. Peripheral blood granulocytes increase significantly and become immature gradually from chronic phase to acceleration phase and to abrupt change phase. Leukemia is a malignant proliferative disease in the hematopoietic system. Any line of leukemia cells proliferates malignantly in bone marrow, and extensive invasion appears in all tissues and organs throughout the body [1, 2]. An abnormal chromosome-Philadelphia (Ph) chromosome occurs among 90% of leukemia patients. Ph chromosome is a breakpoint cluster region (BCR) on the 9^th^ chromosome q34 [3–5]. With the constant deepening of relevant studies on tyrosine kinase inhibitors, dasatinib becomes a first-line drug in the treatment of CML and the first tyrosine kinase inhibitor (TKI). With the continuous development of the second generation of TKI, the second generation BCR-ABL kinase inhibitor dasatinib emerges. Dasatinib is applicable mainly for patients who do not respond to imatinib treatment and shows excellent therapeutic effects on patients [6–8]. However, dasatinib can cause some adverse reactions in treatment. Hemocytopenia is a common adverse reaction in TKI treatment, which could result in water-sodium retention, such as hydrothorax. A few patients suffer from cardiovascular events [9].

Information technology, translation medicine, evidence-based medicine, and pharmacoeconomics are developed rapidly. The study on clinical medicine is greatly advocated by the state, and the demand for science and research is still continuously growing. Traditional statistical methods can only select data surface information, which restricting the generality of experiments. Besides, the function of drugs in real clinical environment cannot be evaluated [10]. With the rise of the new subject of data mining, “big data” process becomes faster and faster. Data mining theory offers the guarantee to the discovery of potential knowledge in big data and supports the long-term care system operation association. Data informatization can effectively manage the information about nursing staff and play certain roles in the analysis and decision-making of government sectors [11–13]. The increasing level of hospital informatization in China provides a platform for big data information analysis. Data mining is widely applied in medical diagnosis, imaging analysis, agricultural environmental engineering, and target recognition [14]. Big data analysis platform is supported by natural language processing, machine learning, and other technologies, and it is implemented in data acquisition, integration, statistics, and analysis, showing significant inherent advantages [15]. Based on hospital data center, the big data analysis platform can form a full disease-specific database with follow-up data, patient data, genomics, and other auxiliary information [16]. Based on machine learning and privacy technical processing, data mart is formed to further explore the correlation between diseases and symptoms by semantic analysis model, knowledge graph, synonym dictionary, and other algorithms. Finally, the application of intelligent in-depth data analysis is realized [17]. The application of data mining is gradually improved, and the obtained results are amazing [18]. Using big data and artificial intelligence technology in the positive promotion of medical data analysis and the improvement of its quality and efficiency becomes a new hot pot.

The cancer recurrence and metastasis may cause immediate death. The molecular markers of cancer recurrence and metastasis can be found by integrated with transcriptomics data from the perspective of system biology, which is of great significance to the prediction and improvement of cancer metastasis and recurrence [19]. In big data analysis platform, massive medical data were acquired and integrated, and computer mining technology was utilized to fuse a large number of multisource and heterogeneous information fusion into standardization to ensure the validity of the subsequent data quality analysis. Besides, gene changes in leukemia were analyzed from the perspective of molecules. The treatment of cancer gene changes in CML by dasatinib was discussed to improve the flexibility and scientific research efficiency of the diagnosis and treatment of cancer and offer a new perspective to the diagnosis and treatment of cancer diseases.

## 2. Materials and Methods

### 2.1. Database

The Online Mendelian Inheritance in Man (OMIM) database is one of the most important bioinformatics databases in molecular genetics at present. Reliable literature sources can ensure the accuracy of data. The data on 625 CML patients and 72 normal people were selected, and the data were divided into a control group and an experimental group. In addition, differential expression analysis was used to recognize differentially expressed genes, and 112 differentially expressed genes (messenger ribonucleic acid (mRNA)) were obtained. Besides, the recognition of differentially expressed genes showed the differences in the gene expression between normal and abnormal samples. After that, the expressed genes were used to recognize target micro-RNA (miRNA) and discover the change mechanism of cancer genes.

### 2.2. Big Data Analysis Platform Architecture

The construction of big data analysis platform was based mainly on medical data, as shown in Figure 1. Electronic case report form (eCRF), genomics, and medical data were supplemented to form medical database. After being sorted out by intelligent data, data mart was formed. Next, structured data analysis was carried out. Semantic analysis model, knowledge graph, and other intelligent algorithms were utilized to explore the potential correlation between diseases and realize the deep application of data. Except for structured data, electronic medical records also contained considerable free text data. Hence, there would be difficulties in analysis, statistics, and search processes. It was significant to adopt intelligent technologies to explore the interesting contents of electronic medical records. Combined with the structural rules in data mining, unique algorithms and models could be refined, and medical mode-based recognition methods were constructed, which laid a foundation for data analysis.

### 2.3. Integrated Gene Expression Analysis System (IEAS)

IEAS mainly provided demand analysis for genomics research data and could improve the input and visualization of large-scale gene expression profiles. Data were preprocessed and then analyzed by the gene expression analysis algorithm. Finally, the complete process of visual and documented output was obtained. The performance of a good operation system platform could offer a complete data mining platform for the gene expression. IEAS design was for the development of large-scale gene expression profile data, which was the core analysis object of software. As the overall framework shown, it was to utilize external data sources to express spectral data and to obtain gene expression matrix after data recognition and processing. On gene expression matrix, the expression mode was queried according to user requirements. According to the specified parameters, the queries were matched in datasets.  Figure 2 displays the data process using IEAS.

### 2.4. Clustering Algorithms

The gene expression analysis algorithm contained in IEAS was utilized for parameters setting, visualization, and file output. Algorithm analysis focused on the data mining of datasets. Clustering was an automatic classification algorithm studying data classification issues and formed the classification mechanism on computers. As a machine learning method, clustering was also included in the concept of data mining with the deepening of relevant studies. Clustering analysis was implemented based on the classification according to the distance and proximity in nature. A set of sample points was added. If function *W* : *Φ* × *Φ*⟶R was called distance function, positive definiteness was expressed by equations (1) and (2) below.

(1) $$\begin{array}{c} W\left(\text{x},y\right)\geq 0, \end{array}$$

(2) $$\begin{array}{c} W\left(\text{x},\text{x}\right)=0. \end{array}$$

Symmetry was expressed by equation (3) below.

(3) $$\begin{array}{c} W\left(\text{x},y\right)=W\left(\text{y},x\right). \end{array}$$

Triangle inequality was expressed by equation (4) below.

(4) $$\begin{array}{c} W\left(\text{x},y\right)+W\left(\text{y},\text{z}\right)\geq W\left(\text{x},\text{z}\right). \end{array}$$

In some cases, equation (4) was reduced to the form of equation (5) as follows.

(5) $$\begin{array}{c} W\left(\text{x},y\right)\leq \max\left(W\left(\text{x},\text{z}\right),W\left(\text{z},y\right)\right). \end{array}$$

There were multiple definitions of the selection of distance in the IEAS system.

Minkowski distance equation was shown as equation (6) below.

(6) $$\begin{array}{c} {\text{s}}_{ij}={\left[\overset{p}{\underset{\alpha =1}{\sum }}{\left|x_{ai}-y_{ai}\right|}^{q}\right]}^{1/q}. \end{array}$$

When *q* = 1, absolute distance equation (Manhattan) was shown as equation (7) below.

(7) $$\begin{array}{c} {\text{s}}_{ij}=\overset{p}{\underset{\alpha =1}{\sum }}\left|x_{ai}-y_{ai}\right|. \end{array}$$

When *q* = 2, Euclidean distance equation (Euclid) was shown as equation (8) below.

(8) $$\begin{array}{c} {\text{s}}_{ij}={\left[\overset{p}{\underset{\alpha =1}{\sum }}{\left|x_{ai}-y_{ai}\right|}^{2}\right]}^{1/2},\text{q}>0. \end{array}$$

When *q* = ∞, Chebyshev distance equation was shown as equation (9) below.

(9) $$\begin{array}{c} {\text{s}}_{ij}=\max\left|x_{ai}-yai\right|. \end{array}$$

In practical application, clustering analysis participated in the whole procedure of the decomposition according to whether there was relevant domain knowledge. Clear tasks were arranged in each procedure.  Figure 3 displays the steps of the clustering algorithm below. Firstly, the features were extracted. After original samples were input, a matrix could be outputted based on the results of feature extraction. A feature index variable was set in each column, and a sample was defined in each row. The feature extraction could have a compact on the analysis of decision-making. The close distance of similar samples in feature space can be obtained by using rational feature extraction schemes. Secondly, the clustering algorithm was executed to mainly obtain the property of “clustering” that could reflect the sample points in *N*-dimensional space. The output in this algorithm was mainly a clustering dendrogram. By the classification from coarse to fine, the specific classification scheme was obtained. Finally, appropriate classification thresholds were selected. In different application scenarios, the selected threshold varied. Domain experts could further analyze the clustering results by using domain knowledge to deepen the understanding of feature points and feature variables.

The clustering algorithm began with putting each individual in its own category, searching for the minimum primitive in distance matrix, and merging the two nearest classes to form a new class. With the diminution of similarities, subclass aggregated into a large category. The definition between classes in the system clustering algorithm would produce different clustering methods. The longest distance method was commonly used to measure the distance among classes. The longest cluster between the samples in two categories was the distance between two categories, and it was expressed by equation (10) below.

(10) $$\begin{array}{c} {\text{s}}_{s}\left(\text{p},q\right)=\max\left\{S_{ij}\left|j\in G_{\text{jk}},j\in G_{\text{q}}\right|\right\}. \end{array}$$

The one party with the shortest distance between the samples in two categories was viewed as the distance between two categories, which was expressed by equation (11) below.

(11) $$\begin{array}{c} {\text{s}}_{CL}\left(\text{p},q\right)=\min\left\{S_{ij}\left|j\in G_{\text{jk}},j\in G_{\text{q}}\right|\right\}. \end{array}$$

The distance between the gravity centers of two categories was seen as the distance between two categories, which was also called center-of-gravity technique. It was expressed by equation (12) below.

(12) $$\begin{array}{c} {\text{s}}_{C}\left(\text{p},q\right)=\text{d}{\bar{x}}_{p}{\bar{x}}_{q}. \end{array}$$

The average distance between the samples in two categories was the distance between two categories, which was also called category average method, which was shown in equation (13) below.

(13) $$\begin{array}{c} {\text{s}}_{G}\left(\text{p},q\right)=\frac{1}{lm}\underset{i\in G_{\text{p}}}{\sum }\underset{j\in G_{\text{q}}}{\sum }d_{ij}. \end{array}$$

The analysis of the variance method was regarded as sum of squares of deviations method, which was expressed by equations (14) and (15) below.

(14) $$\begin{array}{c} {\text{s}}_{\text{p}}=\underset{x_{i}\in G_{\text{p}}}{\sum }\left(x_{i}-{\bar{x}}_{p}\right)\left(x_{i}-{\bar{x}}_{p}\right), \end{array}$$

(15) $$\begin{array}{c} {\text{s}}_{\text{p}}=\underset{x_{i}\in G_{\text{p}}}{\sum }\left(x_{i}-{\bar{x}}_{\text{q}}\right)\left(x_{i}-{\bar{x}}_{q}\right). \end{array}$$

In equations (14) and (15), ${\bar{x}}_{q}$ and ${\bar{x}}_{p}$ referred to gravity centers *G*_*p*_ and *G*_*q*_.*G*_*p*_ and *G*_*q*_ merged into *G*_*r*_, which contained *m* + 1 individuals.

Nanoequation (16) represented sum of squares of deviations as follows.

(16) $$\begin{array}{c} {\text{s}}_{\text{r}}=\underset{x_{r}\in G_{\text{p}}}{\sum }\left(x_{k}-{\bar{x}}_{\text{r}}\right)\left(x_{k}-{\bar{x}}_{\text{r}}\right). \end{array}$$

In equation (16), ${\bar{x}}_{r}$ denoted the gravity center of *G*_*r*_ in the equation and (*S*_*r*_ − *S*_*p*_ − *S*_*q*_) referred to the distance between *G*_*p*_ and *G*_*q*_.

The initial matrices of the several above clustering methods were the same, and the basic procedures were also the same. The summary of a recursive equation would be more useful for computer programming. The gene classes with the highest expression similarity were grouped together to form system clustering trees. The designed gene classes were defined as follows.

In the class of Hierarchy ExpData, ExpressData was needed to be utilized to point to the corresponding gene expression vector. ClusterSzize was used to store the number of all child nodes in the class, and distance was used to store the platform height of the class. Hierarchy ExpData pointed to the left and right child nodes as well as the parent nodes of the nodes. The number of clusters obtained by summing up other variables restored node position.

Entropy and mutual information described the relevance among different genes. The entropy of gene expression mode was the measure of the information contained in the mode. *Q* was used to represent a gene expression mode, and the calculation method of entropy was expressed by equation (17) below.

(17) $$\begin{array}{c} \text{H}\left(\text{Q}\right)=-\overset{\text{n}}{\underset{i=1}{\sum }}P\left(q_{i}\right)\log_{2}\left(P\left(q_{i}\right)\right). \end{array}$$

### 2.5. Implementation of Component Analysis

In IEAS, the implementation of principal component analysis function was based on the analysis of gene expression profiles by samples or gene expression vectors. Firstly, parameters were set to calculate covariance matrix, and then some other indicators were calculated, including characteristic values, feature vectors, and variance contribution rate. After that, principal components were selected, and the visual analysis of the results was carried out. Based on variance contribution rate and cumulative variance contribution rate of vectors, total contribution value was 85%. After the selection of principal components, visual output was conducted.

The experiment was performed in Windows system. The system used Java2 platform and utilized JBuilder8 as the development tool. The language was Mlab7.13 compilation environment, the internal memory was 8G, the main frequency was 3.0GHz, and the processor was Inter with quad core.

### 2.6. Efficacy of Dasatinib in the Treatment of CML

30 patients with advanced CML treated with dasatinib (11 were in accelerated phase, and 19 were in blast phase). Among the 30 patients, 16 were females, and 17 were males, with an age range of 23-61 years old and an average age of 43.41 years old. All patients took dasatinib, which were not minced or sliced. The medications in the 30 patients should be adjusted according to the specific conditions. Complications during the treatment had to be treated timely. All patients insisted on taking the medication for more than 1 month, and the median follow-up time was more than 5 months (1-24 months). The response rate and side effects after taking it were recorded. The efficacy was evaluated based on the management guidelines and efficacy evaluation criteria in 2013 European Leukemia Network (ELN).

### 2.7. Statistical Analysis

Statistics were completed by SPSS17.0, and *P* < 0.05 indicated that there was a significant difference in statistics.

## 3. Results

### 3.1. Gene Difference Analysis

The data on 136 CLM samples, the normal sample data in 61 databases, and the molecular markers between differentially expressed genes and cancer genes were utilized to stratify and cluster the expression progression of 20 differentially expressed genes, so as to assess the relevance between differentially expressed genes and cancer genes. As Figure 4 demonstrated below, cancer samples and normal samples were divided into two different clusters. In other words, 20 differentially expressed genes showed their respective properties between cancer samples and normal samples. The results indicated that the specific differences of 20 gene features were significant.

The selected big data analysis platform was OMIM. CLM genes were analyzed by deoxyribonucleic acid (DNA) sequence recognition regulatory that analyzed the combination of transcription factors.  Figure 5 shows the selection of *n*-tuples. For example, sequence 1 was CGTGAAC, and sequence 2 was ATCGTGA. If the value of *n* was 5, the corresponding matrix was expressed as follows in Figure 5.

### 3.2. Similarity Measurement

Gene expression data mainly came from gene chip, which was utilized to obtain mRNA data of gene transcription results on a large scale. Serial analysis of gene expression (SAGE) and differences displayed a class technology of rapid detection of proteins. Before data clustering, the similarities of the data contained in gene expression matrices were analyzed.  Figure 6 shows the results of similarity measurement below. The two patterns in Figure 6 represent two different gene sequences. A shorter distance indicated more similar modes. On the contrary, differential mode was larger.  Figure 6(a) displays two modes with similar architectural relationships.  Figure 6(b) demonstrates two modes with similar variation trends.  Figure 6(c) presents two gene regulatory modes with similar inputs. However, the results of the regulation were different and even showed an opposite trend.

### 3.3. Principal Component Analysis (PCA)

PCA analysis revealed various results in different experimental conditions.  Table 1 shows the values of principal components corresponding to the experimental conditions of 0.5, 5, 7, 9, and 11.

The left one of Figure 7(a) presented the characteristic values corresponding to different elements, and the right one of Figure 7(b) showed the results of the percentage changes corresponding to different elements. Based on Figure 7, the difference in the variation trends between characteristic values and percentage changes was not obvious. When principal component was 1, characteristic value was the maximum.

### 3.4. Changes of Principal Component Coefficients

As Figure 8 demonstrated below, the change curves of three components were generally consistent, showing a trend of rise followed by decline. The first element coefficient showed a trend of rise followed by decline, and second as well as third one both showed a trend of decline followed by rise.

### 3.5. Gene Expression Features

In cancer genomic maps, mRNA datasets of CML patients were selected, including a total of 120 samples and 20,614 mRNAs. In miRNA datasets, there were 202 samples, including 1,406 miRNAs. 10 miRNAs and 20 mRNAs were screened by miRNA–mRNA regulation template. The gene expression showed that the expression level among CML cases was higher than that in normal control group, and the difference demonstrated statistical meaning.  Figure 9 displays the information about 20 differentially expressed genes below.

### 3.6. Efficacy Analysis

The efficacy analysis results showed that the mortality rate in the accelerated phase was 27.27%, and that in the blast phase was 63.16%. 7 of the 11 patients in the accelerated phase had adverse reactions such as pericardial effusion and fever, and 13 of the 19 patients in the blast phase had adverse reactions such as fever, pleural effusion, and pericardial effusion (Figure 10).

## 4. Discussion

CML is a relatively common hematological malignancy, and the emergence of TKI has changed the treatment process of CML. Dasatinib is a second-generation TKI drug that can inhibit multiple drug-resistant mutations other than T315I, and its inhibitory ability on unmutated BCR/ABL activity is significantly stronger than that of first-generation TKI drugs. In this work, it retrospectively analyzed 3 of 30 patients who were relieved due to systemic bone pain and bone destruction. Among the adverse reactions, bone marrow suppression, fever, and pleural effusion were more common. It may be related to the fact that the patient's primary disease is in the accelerated or blast phase. Dasatinib has good efficacy in the treatment of patients with advanced CML.

Data mining refers to the recognition of useful information from considerable, fuzzy, noisy, incomplete, and random datasets [20]. The main purpose of applying data mining technology in gene analysis is to process massive gene expression profile data by strong analytical capacity, find the relationship networks existing among genes, and provide the basis for the study on gene changes [21, 22]. In Internet hybrid treatment, clinical treatment tests offered considerable data from various sources. The clinical application of relevant modes in the mining of complex data is an arduous task. Rocha et al. [23] supplemented the methods of the search for alternatives to data mining by relevant experimental data and determined the predictive factors used in the system with clinical significance in treatment results. In the big data analysis platform, gene expression data were analyzed to discover the directly risk factors of related diseases and the activity law of relevant genes. In the analysis of gene regulatory networks, a gene network consisted of a group of biomolecules and the interaction among them. These biomolecules could offer some specific cell function tasks. The data were analyzed to represent the gene network, which could describe the function paths in cell tissues [24]. Besides, IEAS was constructed and applied in data mining platform. The system could integrate various analytical methods to obtain the relationship between gene modes in gene expression profiles and look for its biological meaning. Lee et al. [25] analyzed the emotions of social media data based on the sentiment analysis data mining method of machine learning. At confidence level of 95%, variance analysis was used for the statistics and comparison among negative, neutral, and positive emotions. The bar chart, word cloud, phrase, entity, and query analyses were realized in terms of natural language processing-based data mining results. Data mining was used to discuss the treatment of cancer gene changes in CML by dasatinib, and the constructed algorithm model showed excellent effects. In this work, an IEAS was constructed. On the basis of data mining, the clustering algorithm was used to automatically classify the data in the database, and the PCA function was adopted to realize the gene expression vector. The IEAS system could incorporate the gene expression analysis vector of JAVA-related technology it contained, and the generated cluster genes showed similar functions. Clustering algorithms could homogenize data and generate visual cluster heat maps. Under different experimental conditions, there are differences in the analysis results of major elements. IEAS can improve the input and visualization of large-scale gene expression profiles and query the expression patterns based on the user needs on the gene expression matrix. The cluster analysis used in this work classified according to the natural clustering and proximity, showing good classification performance.

Some studies revealed that sox4, RASGRP1, Rasgrp3, IGFIR, IGF2R, CK6, STK38, LEF1, and other cancer genes were of great significance to the prognosis of leukemia. The functional regulatory modules of miRNA and mRNA played certain roles in the development of cancer [26]. The data on 625 CML patients and 72 normal people were selected to obtain 112 differentially expressed genes (mRNA), which was recognized by differential expression analysis to reflect the differences in the gene expression between normal and abnormal samples. After that, these expressed genes were utilized to recognize target miRNA and discover the change mechanism of cancer genes. Further discussion of this study, please refer to references [27–30].

## 5. Conclusion

In this work, an IEAS was constructed, and the data was automatically classified by the online human Mendelian genetic database and clustering algorithm. It was found that the messenger RNA dataset of CML patients was selected from The Cancer Genome Atlas and included 120 samples with a total of 20,614 mRNAs. The data were screened by miRNA-mRNA regulatory templates, and 20 differentially expressed mRNAs were obtained. The constructed genetic analysis system could process large-scale data. The IEAS proposed in this work could mine and analyze the gene expression data. Dasatinib showed a good curative effect in the treatment of CML and had broad application prospects in clinical application. In addition, the clustering analysis and visualization input functions of similar expression patterns also provided a new perspective for future gene expression data mining. In subsequent studies, extended analysis of polygene expression data would be performed on IEAS. In addition, how to quickly filter out the required relevant data from large-scale data was also a hotspot worthy of research. The sample size in this work was small, especially in the accelerated phase; so, it was necessary to expand the study for further discussion.

## Figures and Tables

**Figure 1:** Architecture of big data analysis platform.

**Figure 2:** Data process using IEAS.

**Figure 3:** Clustering algorithm steps.

**Figure 4:** Results of gene difference analysis.

**Figure 5:** Displayed results of two gene sequence matrices.

**Figure 6:** Similarity measurement.

**Figure 7:** Changes of characteristic values corresponding to different elements.

**Figure 8:** Changes of different element coefficients.

**Figure 9:** Analysis of coexpression and differential expression of differentially expressed mRNA.

**Figure 10:** Mortality and adverse effect outcomes.

**Code 1:** 

**Table 1:** PCA.

Experimental conditions	1	2	3	4	5
*N* = 0.5	0.2065	-0.7409	-0.5214	0.2578	0.0654
*N* = 5	0.3946	-0.1152	0.3218	-0.0017	0.5817
*N* = 7	0.5542	0.8231	0.5575	0.4954	-0.1102
*N* = 9	0.4661	0.4571	-0.1528	0.1154	-0.5321
*N* = 10	0.4668	0.3124	-0.4665	-0.5132	0.3218

## Data Availability

The data used to support the findings of this study are available from the corresponding author upon request.

## References

[1] Hochhaus A., Baccarani M., Silver R. T. (2020). European LeukemiaNet 2020 recommendations for treating chronic myeloid leukemia. *Leukemia*.

[2] Hijiya N., Suttorp M. (2019). How I treat chronic myeloid leukemia in children and adolescents. *Blood*.

[3] Jabbour E., Kantarjian H. (2018). Chronic myeloid leukemia: 2018 update on diagnosis, therapy and monitoring. *American Journal of Hematology*.

[4] Cortes J. E., Jimenez C. A., Mauro M. J., Geyer A., Pinilla-Ibarz J., Smith B. D. (2017). Pleural effusion in dasatinib-treated patients with chronic myeloid leukemia in chronic phase: identification and management. *Clinical Lymphoma Myeloma and Leukemia*.

[5] Jabbour E., Kantarjian H. (2020). Chronic myeloid leukemia: 2020 update on diagnosis, therapy and monitoring. *American Journal of Hematology*.

[6] Naqvi K., Jabbour E., Skinner J. (2020). Long-term follow-up of lower dose dasatinib (50 mg daily) as frontline therapy in newly diagnosed chronic-phase chronic myeloid leukemia. *Cancer*.

[7] Cirmi S., El Abd A., Letinier L., Navarra M., Salvo F. (2020). Cardiovascular toxicity of tyrosine kinase inhibitors used in chronic myeloid leukemia: an analysis of the FDA adverse event reporting system database (FAERS). *Cancers (Basel)*.

[8] Cortes J. E., Kim D. W., Pinilla-Ibarz J. (2018). Ponatinib efficacy and safety in Philadelphia chromosome-positive leukemia: final 5-year results of the phase 2 PACE trial. *Blood*.

[9] Talpaz M., Saglio G., Atallah E., Rousselot P. (2018). Dasatinib dose management for the treatment of chronic myeloid leukemia. *Cancer*.

[10] Li J., Xu Q., Cuomo R., Purushothaman V., Mackey T. (2020). Data mining and content analysis of the Chinese social media platform Weibo during the early COVID-19 outbreak: retrospective observational Infoveillance study. *JMIR Public Health and Surveillance*.

[11] Roumani A. M., Madkour A., Ouzzani M., McGrew T., Omran E., Zhang X. (2019). BioNetApp: an interactive visual data analysis platform for molecular expressions. *PLoS One*.

[12] Stephens C. R., Sierra-Alcocer R., González-Salazar C. (2019). SPECIES: a platform for the exploration of ecological data. *Ecology and Evolution*.

[13] Dunn L., Jolly D. (2018). Automated data mining of a plan-check database and example application. *Journal of Applied Clinical Medical Physics*.

[14] Gruendner J., Wolf N., Tögel L., Haller F., Prokosch H. U., Christoph J. (2020). Integrating genomics and clinical data for statistical analysis by using GEnome MINIng (GEMINI) and fast healthcare interoperability resources (FHIR): system design and implementation. *Journal of Medical Internet Research*.

[15] Yu Z., Amin S. U., Alhussein M., Lv Z. (2021). Research on disease prediction based on improved deep FM and IoMT. *IEEE Access*.

[16] Lv Z., Qiao L. (2020). Analysis of healthcare big data. *Future Generation Computer Systems*.

[17] Blatti C., Emad A., Berry M. J. (2020). Knowledge-guided analysis of "omics" data using the KnowEnG cloud platform. *PLoS Biology*.

[18] Julkowska M. M., Saade S., Agarwal G. (2019). MVApp-multivariate analysis application for streamlined data analysis and curation. *Plant Physiology*.

[19] Liang D., Liu Q., Zhou K., Jia W., Xie G., Chen T. (2020). IP4M: an integrated platform for mass spectrometry-based metabolomics data mining. *BMC Bioinformatics*.

[20] Itzel T., Neubauer M., Ebert M., Evert M., Teufel A. (2020). Hepamine - a liver disease microarray database, visualization platform and data-mining resource. *Scientific Reports*.

[21] Sigdel D., Kyi V., Zhang A. (2019). Cloud-based phrase mining and analysis of user-defined phrase-category association in biomedical publications. *JoVE (Journal of Visualized Experiments)*.

[22] Chen W., Gao C., Liu Y., Wen Y., Hong X., Huang Z. (2020). Bioinformatics analysis of prognostic miRNA signature and potential critical genes in colon cancer. *Frontiers in Genetics*.

[23] Rocha A., Camacho R., Ruwaard J., Riper H. (2018). Using multi-relational data mining to discriminate blended therapy efficiency on patients based on log data. *Internet Interventions*.

[24] Yim A., Koti P., Bonnard A. (2020). mitoXplorer, a visual data mining platform to systematically analyze and visualize mitochondrial expression dynamics and mutations. *Nucleic Acids Research*.

[25] Lee M. J., Lee T. R., Lee S. J., Jang J. S., Kim E. J. (2020). Machine learning-based data mining method for sentiment analysis of the Sewol Ferry disaster's effect on social stress. *Frontiers in Psychiatry*.

[26] Zhao J. L., Zhang Z. H., Wang R. (2019). Expression of Transcription Factor SOX4 in Acute Myeloid Leukemia and Its Clinical Significance. *Zhongguo Shi Yan Xue Ye Xue Za Zhi*.

[27] Mohan P., Subramani N., Alotaibi Y., Alghamdi S., Khalaf O. I., Ulaganathan S. (2022). Improved metaheuristics-based clustering with multihop routing protocol for underwater wireless sensor networks. *Sensors*.

[28] Rawat S. S., Alghamdi S., Kumar G., Alotaibi Y., Khalaf O. I., Verma L. P. (2022). Infrared small target detection based on partial sum minimization and total variation. *Mathematics*.

[29] Srilakshmi U., Veeraiah N., Alotaibi Y., Alghamdi S., Khalaf O. I., Subbayamma B. V. (2021). An improved hybrid secure multipath routing protocol for MANET. *Access*.

[30] Mani V., Manickam P., Alotaibi Y., Alghamdi S., Khalaf O. I. (2021). Hyperledger healthchain: patient-centric IPFS-based storage of health records. *Electronics*.

